The article "Prevalence and Risk Factors of Burnout Syndrome during COVID-19 Pandemic among Healthcare Providers in Thailand" was published in 2023. Journal: J Environ Public Health.

# Prevalence and Risk Factors of Burnout Syndrome during COVID-19 Pandemic among Healthcare Providers in Thailand

**DOI:** 10.1155/2023/5719241

**Published:** 2023-05-30

**Authors:** Dujrath Somboonviboon, Yingvitch Wittayawisawasakul, Petch Wacharasint

**Affiliations:** Division of Pulmonary and Critical Care Medicine, Department of Medicine, Phramongkutklao Hospital, Bangkok, Thailand

## Abstract

**Objective:**

To study prevalence, risk factors, and consequences of the COVID-19 pandemic related to Burnout syndrome (BOS) among Thai healthcare providers (HCPs) during the COVID-19 pandemic.

**Methods:**

We performed a cross-sectional study among HCPs, involved in caring for patients during the pandemic in two periods (1st period, May–Jun 2021, and 2nd period, Sep-Oct 2021). Data were distributed using electronic questionnaires. BOS was defined if respondents exhibited a high level of at least one domain in the Maslach Burnout Inventory criteria. The primary outcome was prevalence of BOS.

**Results:**

Altogether, 2,027 and 1,146 respondents were enrolled in the 1st and 2nd periods, respectively. Most respondents were female (73.3, 68.2%). The top three job positions were physicians (49.2, 58.9%), nurses (41.2, 30.6%), and nursing assistants (4.8, 6.5%), respectively. No difference was found in overall prevalence of Burnout syndrome during the 1st and 2nd periods (73 vs. 73.5%, *p*=0.80). Using multivariate analysis, significant risk factors for Burnout syndrome in both periods were (1) living with family (odds ratio (OR) 1.3 and 1.5), (2) tertiary care hospital (OR 1.92 and 2.13), (3) nurse (OR 1.38 and 2.29), (4) nursing assistant (OR 0.92 and 4.81), (5) salary ≤40,000 THB (OR 1.53 and 1.53), (6) >20 patients per shift (OR 1.55 and 1.88), (7) >6 shifts after hours monthly (OR 1.26 and 1.49), and (8) ≤1 rest day weekly (OR 1.3 and 1.4).

**Conclusion:**

We found a high prevalence of Burnout syndrome among Thai HCPs during the pandemic. Knowing those risk factors may provide a strategy to BOS during the pandemic.

## 1. Introduction

Burnout syndrome (BOS) is a work-related stress syndrome described as diminished interest and exhaustion caused by experiencing an inability to cope with emotional stress at work [1, 2]. This syndrome has been frequently associated with specific consequences for individuals (depression, lack of motivation, and workplace violence in a situation mutual with burnout) and also for health institutions (shortage of healthcare providers (HCPs), strain of healthcare systems, malpractice litigation, and poor quality of care) resulting in decreased organization efficiency [3–9]. BOS has been recognized as a psychological problem and has become much more prevalent in the last decade; it was defined as consisting of three qualitative dimensions, namely, emotional exhaustion (EE), depersonalization (DP) or cynicism, and reduced personal accomplishment (PA) [10–13]. BOS develops slowly and could be triggered by multiple factors. However, it has almost never been identified in its early stages [10, 14].

The article "Prevalence and Risk Factors of Burnout Syndrome during COVID-19 Pandemic among Healthcare Providers in Thailand" was published in 2023. Journal: J Environ Public Health.

Before the emergence of coronavirus disease 2019 (COVID-19), the prevalence of BOS among HCPs was found to be between 25 and 62.6% and varied across countries [15–27]. Currently, the global pandemic of COVID-19 has caused numerous infected cases and deaths [28], a rapidly increasing number of patients, high workload, shortage of medical resources, the pain of losing patients and colleagues, and the risk of infection for themselves and their families may cause more BOS among HCPs, but the effect of the pandemic on BOS is yet poorly understood. Therefore, this study aimed to evaluate the prevalence and risk factors of BOS among HCPs during the COVID-19 pandemic in Thailand.

## 2. Methods and Materials

### 2.1. Participants

We conducted a cross-sectional analytic study among HCPs (physicians, nurses, nursing assistants, pharmacists, laboratory staff, and radiology staff) during the COVID-19 pandemic in Thailand. Based on social distancing policy during the COVID-19 pandemic, participants were recruited through online social media platforms (Google Forms) using a snowball technique. The inclusion criteria included full-time employees at all types of medical centers in Thailand, including university hospitals, tertiary center hospitals, secondary center hospitals, community hospitals, private hospitals, and private clinics, who were willing to answer a questionnaire. Either general medical centers or specialized COVID-19 centers were included in this study. Exclusion criteria included (1) under 20 years of age and (2) not consenting to a questionnaire. This study was approved by the Ethics Board of the Royal Thai Army Medical Department (R075q/64_Exp) and all participants voluntarily signed the consent form before joining the study.

### 2.2. Data Collection

Firstly, we conducted a cross-sectional analytic study from May 1, 2021, to June 30, 2021. Following our data analysis, the number of patients hospitalized with COVID-19 dramatically increased (May 31, 2021, totaled 50,416 patients while September 30, 2021, totaled 116,075 patients) as reported by the Center for COVID-19 Situation Administration (CCSA) [29]. Therefore, to compare and analyze whether more COVID-19 hospitalized cases increased the prevalence of BOS, we decided to continue collecting data from September to October 2021. We defined the data during May 1 to June 30, 2021, as the 1st period while data from September 1 to October 31, 2021, were classified as the 2nd period. We also tested whether risk factors for BOS during the first period were also replicated during the second period.

The article "Prevalence and Risk Factors of Burnout Syndrome during COVID-19 Pandemic among Healthcare Providers in Thailand" was published in 2023. Journal: J Environ Public Health.

### 2.3. Questionnaire

This study was conducted using a Thai language electronic survey-based questionnaire consisting of five parts: (i) demographic data, (ii) personal information, (iii) work characteristics, (iv) consequences related to COVID-19, and (v) Maslach Burnout Inventory (MBI) Human Service survey. Thus, we collected gender, age, current marital status (single, married, and divorce), and accommodation status (single living, living with family, and living with colleague/friend). In terms of the work characteristics, participants were required to verify their type of workplace (university hospital, tertiary center hospital, secondary center hospital, community hospital, private hospital, private clinic, or others), job position (physician, nurse, nursing assistant, pharmacist, laboratory staff, radiologic staff, administrative staff, or others), type of specialist, work experience duration, range of monthly income, and current workload including the number of patients, work hours, and days off. Regarding the consequences of COVID-19 pandemic related to BOS, the questionnaires comprised workload, position change, concerns of family health, and exhaustion from using personal protective equipment. The consequences of COVID-19 pandemic related to BOS were verified if the participants responded “yes” to the following questions: “Is your workload heavier?” “Have you had to change your job to less satisfactory one?” “Do you have any concerns about your health?” “Do you have any concerns about your family's health?” “Do you find it difficult to live in your daily life in the COVID-19 pandemic?” “Are you exhausted from wearing personal protective equipment (PPE) whilst caring COVID-19 patients?”.

As it is considered an internationally acknowledged and validated instrument for measuring job burnout, MBI Human Services Survey is a 22-item questionnaire, in which the answers are self-graded frequency score from 0 (never) to 6 (every day). All 22 questions are categorized in 3 dimensions, including EE, DP, and PA. The summation for each aspect is stratified as high, average, or low. BOS is defined if the participants revealed high EE, high DP, or low PA [30–34]. The MBI Human Service survey has previously been translated into Thai and has been well tested for reliability with Cronbach's alpha coefficients for EE of 0.92, DP of 0.66, and PA of 0.65 [35, 36].

### 2.4. Statistical Analysis

According to the related study of BOS during the COVID-19 pandemic conducted by Nishimura et al. [37], adequate sample size in our study must comprise at least 385 participants.. Primary outcome was prevalence of the BOS in HCPs during the COVID-9 pandemic. Secondary outcomes consisted of risk factors for the BOS and consequences of the COVID-19 pandemic related to BOS. Descriptive statistics, including percentage, frequency, average, and standard deviation, were used to demonstrate the demographic data and prevalence of BOS. To analyze risk factors for BOS, we performed univariate comparison first then constructed multivariate regression analysis. Inferential statistics were used by exhibiting a statistical significance at alpha of 0.05, including Pearson's chi-square test and independent-student *t*-test.

The article "Prevalence and Risk Factors of Burnout Syndrome during COVID-19 Pandemic among Healthcare Providers in Thailand" was published in 2023. Journal: J Environ Public Health.

## 3. Results

### 3.1. Respondent Characteristics

Exactly 2,027 and 1,146 respondents in were enrolled the 1st and 2nd periods, respectively. Most were physicians (49.2, 58.9%), followed by nurses (41.2, 30.6%) and nursing assistants (4.8, 6.5%).

### 3.2. Baseline Characteristics of Respondents in Both Periods

Most respondents were female (73.3, 68.2%), single status (60.3, 67.1%), and living with their families (56.2, 50.9%). Most worked at the universal hospitals (41.9, 37.6%) with working experience between 6 and 10 years (28.9, 36.6%) and most had a salary between 20,001 and 30,000 THB (24.9, 25.7%) (Table 1).

### 3.3. Prevalence of BOS

Although the overall prevalence of BOS was high in both study periods, no difference was found in overall prevalence of BOS between the 1st (73%) and the 2nd period (73.5%) (*p*=0.8). In the 1st and 2nd periods, participants experienced BOS at a high EE of 51.3 and 49%, high DP of 24.6 and 27.1%, and high level of decreased PA of 47.9 and 51.5%, respectively (Table 2). Physicians working in the 1st period experienced more BOS than physicians working in the 2nd period (71.3 vs. 66.8%, *p*=0.015), while the nurses and nursing assistants working in the 1st period experienced less BOS than the nurses (74.9 vs. 82.3%, *p*=0.013) and nursing assistants (69.1 vs. 90.7%, *p*=0.002) working in the 2nd period (Figure 1). In the subgroup analysis based on physician specialty, no difference was found in the prevalence of BOS between the two study periods, except among other specialties (Figure 2).

In the 1st period, of 997 physicians, 71.3% experienced BOS, from high EE of 47.1%, high DP of 28.1%, and high level of decreased PA of 50.2%. Of 836 nurses, 74.9% experienced BOS, from high EE of 58%, high DP of 21.4, and high level of decreased PA of 42.6%. Of 97 nursing assistants, 69.1% experienced BOS, from high EE of 47.4%, high DP of 11.3%, and high level of decreased PA of 59.8%.

The article "Prevalence and Risk Factors of Burnout Syndrome during COVID-19 Pandemic among Healthcare Providers in Thailand" was published in 2023. Journal: J Environ Public Health.

In the 2nd period, of 675 physicians, 66.8% experienced BOS, from high EE of 44.1%, high DP of 30.8%, and high level of decreased PA of 49%. Of 351 nurses, 82.3% experienced BOS, from high EE of 60.1%, high DP of 23.4%, and high level of decreased of PA 51.6%. Of 75 nursing assistants, 90.7% experienced BOS, from high EE of 44%, high DP of 20%, and high level of decreased PA of 69.3%.

### 3.4. Risk Factors for BOS

Using multivariate analysis, the risk factors for BOS in both periods included (1) living with family (odds ratio (OR) = 1.3 and 1.5; *p*=0.037 and 0.02), (2) working in a tertiary care hospital (OR = 1.92 and 2.13; *p*=0.007 and  < 0.001), (3) nurse position (OR = 1.38 and 2.29; *p*=0.008 and  < 0.001), (4) nursing assistant position (OR = 0.92 and 4.81; *p*=0.719 and  < 0.001), (5) earning salary ≤40,000 THB (OR = 1.53 and 1.53; *p* < 0.001 and 0.002), (6) having >20 patients per shift (OR = 1.55 and 1.88; *p* < 0.001 and  < 0.001), (7) working >6 shifts after hours monthly (OR = 1.26 and 1.49; *p*=0.026 and 0.004), and (8) having ≤1 rest day weekly (OR = 1.3 and 1.4; *p*=0.012 and 0.018) (Table 3).

### 3.5. Consequences of COVID-19 Pandemic Related to BOS

Using multivariate analysis, consequences of COVID-19 pandemic related to BOS were heavier workload, unsatisfied job, personal and family health concerns, difficulty in daily life, and exhaustion of wearing personal protective equipment (all *p* < 0.05 in both periods) (Table 4).

## 4. Discussion

This study demonstrated a high prevalence of BOS in HCPs during the COVID-19 pandemic in Thailand. We found a high prevalence of BOS in both periods of the study (73.0 and 73.5%). Compared to a previous study before the COVID-19 pandemic, the prevalence of BOS among Thai ICU physicians and nurses was 65.15 and 60.95%, respectively [23] while a previous systematic review during the COVID-19 pandemic, the pooled overall BOS prevalence was 52% (95% CI 40–63%) [38]. We also found that the major domain contributing to BOS was high EE in the 1st period and high level of decreased PA in the 2nd period. These findings were aligned to a previous study which found that most of Italian HCPs experienced high EE and decreased PA during the COVID-19 pandemic [39].

Physicians in our study experienced lower BOS in the 2nd period but varied between specialties. Although it did not achieve statistical significance, pulmonologists and pediatricians seem increased prevalence of BOS in the 2nd period. The possible explanations may be most severe COVID-19 cases were taken care by pulmonologists. Increasing numbers of patients have may put more severe cases as well as higher workload on the pulmonologists. Likewise, a greater number of children with COVID-19 infection in the 2nd period may have contributed to higher pediatrician workloads. The nurses and nursing assistants dealing with a higher prevalence of BOS in the 2nd period may have possibly been due to more hospitalized COVID-19 cases in the 2nd period of the study and the increased burden of nursing care.

The article "Prevalence and Risk Factors of Burnout Syndrome during COVID-19 Pandemic among Healthcare Providers in Thailand" was published in 2023. Journal: J Environ Public Health.

The risk factors for BOS we found in our study included (1) living with family, (2) working in a tertiary care hospital, (3) nurse position, (4) nursing assistant position, (5) earning salary ≤40,000 THB, (6) having >20 patients per shift, (7) having >6 shifts after hours monthly, and (8) having ≤1 rest day weekly. These important findings provide public health strategies to prevent BOS in HCPs during the COVID-19 pandemic. Even though workload is an uncontrollable factor during the pandemic, organizations need to ensure adequate staging through ongoing evaluation of workloads. Optimization of professional rewarding systems, including salaries and motivational support such as temporary accommodation or family welfare, should also be considered. Although the role of family relations may be less pronounced than job satisfaction itself, some studies found that families can take some action in the mitigation of occupational BOS in HCPs [26, 40, 41]. In contrast, our study found that living with family during the pandemic increased the risk of BOS. This finding is possibly explained by the concern of family members becoming infected through HCPs. A previous study in Indian HCPs during the COVID-19 pandemic [42] used a questionnaire to evaluate BOS. They found that 50% of participants had a statistically significant concern and reported exhaustion from working during the pandemic. Those authors also worried about becoming infected and transmitting the disease to their families. One more risk factor for BOS in our study was working in a tertiary care hospital; a possible explanation why working in the tertiary care hospitals increased risk of BOS may be because of receiving very severe cases from other hospitals which have less facility. Also, inappropriate ratios of HCPs to number of patients as well as insufficient medical equipment compared to the number of patients may play a major role to BOS. Other risk factors such as low salary, increased workload, and less rest days weekly also increased risk for BOS because these factors might reduce motivation to work.

Compared to previous studies, this study revealed novel findings. We demonstrated that the COVID-19 pandemic is directly linked to BOS through both physical and mental drawbacks. For example, we found that HCPs with BOS were significantly exhausted from wearing PPE whilst caring for COVID-19 patients, and had more concerns about their and their family's health. Providing several specific preventive interventions during a pandemic may be a key to potential BOS reduction, including measures such as confirmation of correct PPE usage, emphasizing ways to reduce the risk of infection, supplying adequate antigen test kits for early detection, and providing isolated accommodation whilst on duty.

The article "Prevalence and Risk Factors of Burnout Syndrome during COVID-19 Pandemic among Healthcare Providers in Thailand" was published in 2023. Journal: J Environ Public Health.

The strengths of our study were a large number of participants with various job positions and various hospital levels in Thailand. This allows our data to be more diverse. We also validated possible risk factors for BOS and consequences of COVID-19 pandemic related to BOS using the 2nd period cohort as a validation cohort with the multivariate analysis. However, our study encountered several limitations. Firstly, respondents in both periods of the study differed which may have affected the comparison of results. Secondly, response bias may have occurred comprising their personal data. Lastly, our data must be carefully interpreted because of heterogeneity in job positions, types of hospital, and various differences in baseline characteristics (i.e., marital status and monthly income).

The finding of high prevalence of BOS in our study may reflect overall growing disappointment in healthcare systems, which need urgent attention because it may result in mental health problems, decreased quality of life among HCPs, and poorer healthcare outcomes [43, 44]. Moreover, preventive interventions, including occupational health surveillance and workplace health promotion programs, should be reviewed for prevention, early diagnosis and therapy of BOS, as well as other pandemic stress-related consequences such as posttraumatic stress disorder and suicide [45–48]. The issue of long-term BOS and mental health problems among HCPs should be examined further and big data intelligence in COVID-19 pandemic may play an important role for further research [49].

## 5. Conclusion

We found a high prevalence of BOS among Thai HCPs during the COVID-19 pandemic. This needs more attention, preventive intervention, and increased public health awareness to reduce BOS in HCPs. Increased workload with low compensation is a major risk factor for BOS. In addition, consequences of COVID-19 pandemic significantly related to BOS among HCPs.

## Figures and Tables

**Figure 1:** Prevalence of Burnout syndrome classified by job positions in both periods. ^*∗*^depicts *p* < 0.05, analysis using the Mann–Whitney *U* test.

**Figure 2:** Prevalence of Burnout syndrome classified by physician specialties. White and black bar graphs represent prevalence of Burnout syndrome (BOS) in the 1st and 2nd periods, respectively. Numbers inside the bar graphs represent the total number of respondents in each physician's specialty. Two dash lines represent average BOS in the 1st (71%) and 2nd periods (67%), respectively. ^*∗*^depicts *p* < 0.05, data analysis using the Pearson chi-square test. CCM: critical care medicine; Pulmo: pulmonologist; ID: infectious disease physician; EM: emergency medicine; Anesth: anesthesiologist; Med: internal medicine; Sx: general surgery; Eye: ophthalmologist; ENT: otolaryngologist; Ped: pediatrician; ^a^Others: physical medicine and rehabilitation physician/obstetrician/radiologist/family medicine physician/pathologist/psychiatrist.

The article "Prevalence and Risk Factors of Burnout Syndrome during COVID-19 Pandemic among Healthcare Providers in Thailand" was published in 2023. Journal: J Environ Public Health.

**Table 1:** Characteristics of respondents in both periods of the study.

Characteristics	1st period (May–Jun)	2nd period (Sep–Oct)
	*N* = 2027	*N* = 1146
*Sex, no (%)*		
Male	524 (25.9%)	359 (31.3%)
Female	1486 (73.3%)	782 (68.2%)
Others	17 (0.8%)	5 (0.4%)

*Age, no (%)*		
<30 years	476 (23.5%)	330 (28.8%)
30–39 years	902 (44.5%)	592 (51.7%)
40–49 years	446 (22%)	161 (14%)
50–59 years	196 (9.7%)	63 (5.5%)
≥60 years	7 (0.3%)	0 (0%)

*Status, no (%)*		
Single	1222 (60.3%)	769 (67.1%)
Marriage	760 (37.4%)	351 (30.6%)
Divorce	46 (2.3%)	26 (2.3%)

*Accommodation, no (%)*		
Single living	497 (24.5%)	329 (28.7%)
Living with family	1139 (56.2%)	583 (50.9%)
Living with a colleague (dormitory)	391 (19.3%)	234 (20.4%)

*Hospital level, no (%)*		
University hospital	849 (41.9%)	431 (37.6%)
Tertiary center hospital (>500 beds)	130 (6.4%)	257 (22.4%)
Secondary center hospital (201–500 beds)	586 (28.9%)	113 (9.9%)
Secondary center hospital (121–200 beds)	78 (3.8%)	86 (7.5%)
Community hospital (10–120 beds)	159 (7.8%)	152 (13.3%)
Private hospital	206 (10.2%)	98 (8.6%)
Private clinic	17 (0.8%)	5 (0.4%)
Others	0 (0%)	3 (0.3%)

*Job position, no (%)*		
Physician	997 (49.2%)	675 (58.9%)
Nurse	836 (41.2%)	351 (30.6%)
Nursing assistant	97 (4.8%)	75 (6.5%)
Pharmacist	73 (3.6%)	7 (0.6%)
Laboratory staff	15 (0.7%)	8 (0.7%)
Radiologic staff	4 (0.2%)	1 (0.1%)
Administrative staff	1 (0.05%)	6 (0.5%)
Others	4 (0.2%)	23 (2%)

*Specialty, no (%)*		
Critical care	222 (11%)	81 (7.1%)
Pulmonology	110 (5.4%)	52 (4.5%)
Infectious disease	55 (2.7%)	44 (3.8%)
Emergency	182 (9%)	88 (7.7%)
Anesthesia	0 (0%)	62 (5.4%)
General medicine	635 (31.3%)	458 (40%)
Surgery	281 (13.9%)	104 (9.1%)
Pediatric	79 (3.9%)	45 (3.9%)
Others	1041 (51.4%)	187 (16.3%)

*Work experience, no (%)*		
<1 years	46 (2.3%)	23 (2%)
1–5 years	428 (21.1%)	331 (28.9%)
6–10 years	585 (28.9%)	420 (36.6%)
11–15 years	368 (18.2%)	171 (14.9%)
16–20 years	191 (9.4%)	81 (7.1%)
>20 years	409 (20.2%)	120 (10.5%)

*Monthly income, no (%)*		
<10,000 THB	34 (1.7%)	14 (1.2%)
10,001–20,000 THB	260 (12.8%)	165 (14.4%)
20,001–30,000 THB	504 (24.9%)	295 (25.7%)
30,001–40,000 THB	403 (19.9%)	235 (20.5%)
40,001–50,000 THB	250 (12.3%)	132 (11.5%)
>50,000 THB	486 (24%)	258 (22.5%)

*Average number of patients monthly, no (%)*		
<20	203 (10%)	102 (8.9%)
21–40	416 (20.5%)	237 (20.7%)
41–60	286 (14.1%)	202 (17.6%)
61–80	181 (8.9%)	104 (9.1%)
81–100	201 (9.9%)	101 (8.8%)
>100	740 (36.5%)	400 (34.9%)

*Average number of patients per shift, no (%)*		
<10	735 (36.3%)	404 (35.3%)
11–20	595 (29.4%)	310 (27.1%)
21–30	274 (13.5%)	151 (13.2%)
31–40	119 (5.9%)	94 (8.2%)
41–50	77 (3.8%)	57 (5%)
>50	227 (11.2%)	130 (11.3%)

*Number of shifts after hours monthly, no (%)*		
0	401 (19.8%)	200 (17.5%)
1–2	175 (8.6%)	92 (8%)
3–4	258 (12.7%)	137 (12%)
5–6	242 (11.9%)	173 (15.1%)
>6	951 (46.9%)	544 (47.5%)

*Average number of rest days weekly, no (%)*		
0–1	830 (40.9%)	492 (42.9%)
2	887 (43.8%)	450 (39.3%)
3	146 (7.2%)	110 (9.6%)
4	92 (4.5%)	47 (4.1%)
5	72 (3.6%)	47 (4.1%)

The article "Prevalence and Risk Factors of Burnout Syndrome during COVID-19 Pandemic among Healthcare Providers in Thailand" was published in 2023. Journal: J Environ Public Health.

**Table 2:** Prevalence and severity of BOS in both periods of the study.

Variables	1st period (May–Jun)	2nd period (Sep–Oct)	*p* value
	*N* = 2027	*N* = 1146	
Burnout syndrome (BOS)	1481 (73%)	842 (73.5%)	0.80

*Emotional exhaustion (EE)*			
Low + average	987 (48.7%)	585 (51%)	0.31
High	1040 (51.3%)	561 (49%)	

*Depersonalization (DP)*			
Low + average	1528 (75.4%)	835 (72.9%)	0.17
High	499 (24.6%)	311 (27.1%)	

*Decreased personal accomplishment (PA)*			
Low + average	1056 (52.1%)	556 (48.5%)	0.006
High	971 (47.9%)	590 (51.5%)	

**Table 3:** Multivariate analysis of risk factors for BOS in both periods of the study.

Variables	1st period (May–Jun)			2nd period (Sep–Oct)		
	Odds ratio	95% CI	*p* value	Odds ratio	95% CI	*p* value
*Age (years)*						
<30	Reference	1	1	Reference	1	1
≥30	0.89	0.58–1.38	0.612	1.48	0.87–2.52	0.145

*Sex*						
Male	Reference	1	1	Reference	1	1
Female	1.06	0.84–1.32	0.629	1.1	0.79–1.52	0.584

*Status*						
Marriage	Reference	1	1	Reference	1	1
Divorce	0.98	0.7–1.36	0.907	1.16	0.77–1.74	0.488
Single	0.88	0.66–1.16	0.353	1.28	0.9–1.81	0.173

*Accommodation*						
Single living	Reference	1	1	Reference	1	1
Living with family	**1.3**	**1.02–1.67**	**0.037**	**1.5**	**1.07–2.12**	**0.019**
Living with colleague (dormitory)	1.03	0.54–1.97	0.934	1.59	0.61–4.11	0.343

*Hospital level*						
University hospital	Reference	1	1	Reference	1	1
Tertiary center hospital	**1.92**	**1.2–3.07**	**0.007**	**2.13**	**1.44–3.15**	**<0.001**
Secondary center hospital	1.57	1.22–2.01	<0.001	1.26	0.79–2.02	0.331

*Job positions*						
Physician	Reference	1	1	Reference	1	1
Nurse	**1.38**	**1.09–1.75**	**0.008**	**2.29**	**1.61–3.27**	**<0.001**
Nursing assistant	0.92	0.57–1.47	0.719	**4.81**	**2.14–10.78**	**<0.001**

*Salary (THB)*						
>40,000	Reference	1	1	Reference	1	1
≤40,000	**1.53**	**1.25–1.87**	**<0.001**	**1.53**	**1.16–2.02**	**0.002**

*Average number of patients per shift*						
≤20	Reference	1	1	Reference	1	1
>20	**1.55**	**1.25–1.93**	**<0.001**	**1.88**	**1.41–2.52**	**<0.001**

*Number of shifts after hours monthly*						
≤6	Reference	1	1	Reference	1	1
>6	**1.26**	**1.03–1.55**	**0.026**	**1.49**	**1.13–1.97**	**0.004**

*Average number of rest days weekly*						
>1	Reference	1	1	Reference	1	1
≤1	**1.30**	**1.06–1.61**	**0.012**	**1.40**	**1.06–1.85**	**0.057**

Statistical significance, *p* value <0.05 was considered as bold values.

The article "Prevalence and Risk Factors of Burnout Syndrome during COVID-19 Pandemic among Healthcare Providers in Thailand" was published in 2023. Journal: J Environ Public Health.

**Table 4:** Multivariate analysis for consequences of COVID-19 pandemic related to BOS in both periods of the study.

Variables	1st period (May–Jun)			2nd period (Sep–Oct)		
	Odds ratio	95% CI	*p* value	Odds ratio	95% CI	*p* value
*Is your workload heavier?*						
No	Reference	1	1	Reference	1	1
Yes	2.97	2.34–3.78	<0.001	3.76	2.73–5.18	<0.001

*Have you had to change your job to less satisfactory one?*						
No	Reference	1	1	Reference	1	1
Yes	2.31	1.79–3.0	<0.001	1.87	1.38–2.53	<0.001

*Do you have any concerns about your health?*						
No	Reference	1	1	Reference	1	1
Yes	2.02	1.6–2.55	<0.001	2.26	1.6–3.2	<0.001

*Do you have any concerns about your family's health?*						
No	Reference	1	1	Reference	1	1
Yes	1.73	1.41–2.12	<0.001	2.02	1.54–2.65	<0.001

*Do you find it difficult to live in your daily life in the COVID-19* ^*a*^ * pandemic?*						
No	Reference	1	1	Reference	1	1
Yes	3.02	2.3–3.96	<0.001	3.38	2.27–5.04	<0.001

*Are you exhausted from wearing personal protective equipment (PPE) whilst caring COVID-19* ^*a*^ * patients?*						
No	Reference	1	1	Reference	1	1
Yes	3.25	2.6–4.06	<0.001	3.21	2.36–4.36	<0.001

^a^COVID-19: coronavirus disease 2019.

## Data Availability

The data that support the findings of this study are available on request from the corresponding author. The data are not publicly available because of privacy or ethical restrictions.

## Abbreviations

BOS: Burnout syndrome
CCSA: Center for COVID-19 situation administration
COVID-19: Coronavirus disease 2019
DP: Depersonalization
EE: Emotional exhaustion
HCPs: Healthcare providers
MBI: Maslach Burnout Inventory
OR: Odds ratio
PA: Personal accomplishment
PPE: Personal protective equipment.
